# A Simulation Analyzing Approach to Estimating the Probability of Airborne Infection Risks in Railway Station Platform Coupling with the Wells-Riley Model and Pathfinder Model

**DOI:** 10.1155/2021/6066109

**Published:** 2021-12-21

**Authors:** Yi-Zheng Dai, Yan-Jiao Chen, Chen-Yang Zhang

**Affiliations:** ^1^School of Architecture, Southeast University, Nanjing, China; ^2^Shanghai Research Institute of Acupuncture and Meridian, Shanghai University of Traditional Chinese Medicine, Shanghai, China

## Abstract

Railway station platforms present a particular challenge, especially during a train departure or arrival where some passengers may have potential conditions that make them vulnerable to airborne infections due to the high density and close proximity of passengers. This study presented a simulation analyzing approach to estimating the probability of airborne infection risks in station platform spaces coupling with the Wells-Riley model and Pathfinder model. We examine the impact of overcrowded area of the station platform on infection rates under various traces of evacuation. The result of the potential risk for three modes is discussed, and the results of the standard model under the same parameter setting are optimised. Next, the impact of the ventilated volume based on uneven distribution of individuals and the exposure time based on evacuation on the infection risk in platform spaces are studied. The relationship between platform spaces overcrowding and the infection risk provided further insights to observe the supporting information.

## 1. Introduction

Many infectious diseases are known to be transmitted via an airborne route, including coronavirus disease (COVID-19) [1], severe acute respiratory syndrome, influenza A virus subtype H1N1 [2], and tuberculosis [3]. Airborne infections pose a particular threat to susceptible individuals whenever they are placed together with the index case in confined spaces [4]. The risk of airborne transmission has been shown to be directly related to the number of susceptible individuals in many population studies [5]. Person-to-person transmission primarily occurs via a direct contact or through droplets spread by coughing, sneezing, talking, and breathing from an infected individual [6]. These infected droplets, containing virus that can remain viable on surfaces for days in favourable atmospheric conditions, can spread 1-2 m and deposit on surfaces [7].

The transmission of infectious diseases can be very rapid in confined spaces, such as prisons, nursing homes, chronic care conditions, detoxification centres, refugee camps, hospitals, and schools with transmission occurring in situations where infected persons are in close contact with others [8]. However, studies addressing station platforms are scarce. Station platforms present a particular challenge, especially during a train departure or arrival where some passengers may have potential conditions that make them vulnerable to infections due to the high density and close proximity of passengers. The majority of the urban population relies on high-speed railways for travel and business purposes [9]. Therefore, it is important to understand the potential infection risks faced by susceptible individuals on station platforms [10].

Although there have been many reports of infectious disease transmission in confined spaces, most of these works have focused on analyzing the relationship among the quanta production rate [11], ventilation mode [12], and exposure duration of the source cases [13]. By comparison, very little work has been undertaken to quantify the risk of airborne transmission with overcrowding in confined spaces. Overcrowding in platform spaces manifests as evacuation of passengers during the departure or arrival phase [14]. Regions with high and low infectious droplet concentrations will simultaneously exist within the same confined space, with the highest concentrations usually occurring close to overcrowded areas. Consequently, the variation of overcrowded areas in platform spaces reflects the effects of passengers' movements on the distribution of the infectious agent throughout the confined spaces during evacuation.

Our objectives were to quantify the impact of overcrowded areas, where infected droplets and air are well mixed compared with the entire platform, on infection rates. A simulation approach is suitable for this study due to the uncertainty of passenger activity trajectories. We optimised the Wells-Riley mathematical model based on a simulation approach of building science to estimate (1) the ventilated volume of an overcrowding area and its variability in platform spaces, (2) the exposure time of passengers during the departure or arrival phase, and (3) the risk for infections in various modes of evacuation to study the relationships between the individual distribution of overcrowding during evacuation and the infection risk in platform spaces.

## 2. Methodology

### 2.1. Study Design

Modelling approaches in building science have focused on the relationship between the human behaviour and spatial layout. Various spatial analysis softwares have been developed in building science and divided into two types: simulation model and sketch model. The simulation model consists of Pathfinder, Ecotect, and Phoenics. These simulation models can perform an interactive analysis based on a three-dimensional space, simulating the influence of factors. The sketch model includes models, such as SketchUp, Revit, 3Ds Max, and AutoCAD. However, these models directly face the creative process of design, and an interactive analysis is often neglected.

The Wells-Riley mathematical model has been used to estimate the airborne infection risk in a confined space [15]. In this model, it is assumed that the air in a room space is completely mixed and that the infectious agent is evenly distributed throughout the room space. In an uneven distribution of passengers due to overcrowding in a platform space, the result will be more accurate only if it is closer to the above assumption state. Coupling building science model and the Wells-Riley model can be a promising means to simulate a confined environment that accomplishes the goals of improving the accuracy of risk results by further optimising a spatial analysis. In this study, Pathfinder was selected because it can track the routes of each occupant and define his or her response to the incident by considering typical behaviours [16].

### 2.2. Volume of a Ventilated Space

In the study, a three-dimensional station platform with a dimension of 450 × 12 × 4 m was selected as the base condition space, and it meets the platform configuration standards of China's high-speed railway stations.  Figure 1 shows the base condition space, which contained two entrance stairs (NS1-NS2), two entrance escalators (NE1-NE2), two exit stairs (XS1-XS2), two exit escalators (EE1-EE2), 20 departure carriage doors (DD1–DD20), and 20 arrival carriage doors (AD1–AD20). Each entrance and exit stair was 18 m long × 3 m wide. Each entrance and exit escalator was 18 m long × 1.2 m wide. Each carriage door was 2.4 m high × 1 m wide.

The station platform is a closed spatial environment without the application of a ventilation system, which eliminates the interference of other factors. The stereo area occupied by a single passenger was called the basic exposure cell (BEC) and denoted by BEC_*i*_ (*i* = 1, 2,…, *n*) [17]. BEC can be divided into several sizes along the width of the human body in the range of *W* = 0.6–1.0 m, as shown in Figure 2, based on different luggage carried by the passengers. BEC is a suitable surrogate volume of exhaled droplet nuclei for studying airborne transmission in a built environment [18]. The volume of ventilated space within the Wells-Riley mathematical model, representing the indoor spatial volume where infected droplets and air were well mixed, was assumed as a stereo area occupied by the passengers in the platform space in this study.

The volume of the ventilated space $\bar{V_{i}}\left(t\right)$ at time *t* is suggested to be calculated by

(1) $$\begin{array}{c} \bar{V_{i}}\left(t\right)=\sum_{i=1}^{n}{\text{BEC}}_{i}\left(t\right), \end{array}$$

where BEC_*i*_ is the sum of the volume occupied by passengers 1 to *i*, *t* is the exposure time during evacuation, *n* is the number of passengers, and $\bar{V_{i}}\left(t\right)$ is the volume of ventilated space at time *t*.

### 2.3. Simulation Modelling

As station platforms are repetitive in the plane and there is no mutual interference between adjacent platforms, it is reasonable and feasible to select a representative case for simulation, as shown in Figure 1. Space boundaries and passenger behaviour are the main factors that can greatly affect the passengers' distribution of overcrowding.  Figure 3 shows the data collected using Pathfinder, which show the geographical pathway of the evacuation that occurred at 1-2 m distance among the passengers. The trajectory of each individual and their response to the environmental stimulation were traced by considering their personal behaviours [17]. The mathematical form of the evacuation process can be written as follows:

(2) $$\begin{array}{c} F_{t}=\left\{U\left(t\right),M\right\}, \end{array}$$

where *F*_*t*_ is a parameter vector *U* (*t*) and a grid matrix *M* with coordinate information (*x*, *y*). The grid matrix *M* provided a reasonable spatial discrete form to quantify the individual distribution, as given by

(3) $$\begin{array}{c} M=\left\{\left(x,y\right)|x_{\text{min}}<x<x_{\max},y_{\min}<y<y_{\max}\right\}. \end{array}$$

Parameter vector *U* (*t*) can be expressed as

(4) $$\begin{array}{c} U\left(t\right)=\left(U_{t1},U_{t2},\ldots ,U_{tn}\right), \end{array}$$

where *U* (*t*) describes the location and velocity of all BEC for each time step in the platform space.

The evacuation process was simulated from time *t*_1_ to *t*_*n*_ using Pathfinder to obtain data on the passenger space-time distribution. The evacuation process calculates the location of BEC by a Lagrangian approach as follows:

(5) $$\begin{array}{c} F_{t}=\left\{\begin{array}{c} x\left(m,t+1\right)=x\left(m,t\right)+U_{tn}\Delta X,\\ y\left(m,t+1\right)=y\left(m.t\right)+U_{tn}\Delta Y, \end{array}\right. \end{array}$$

where *m* is the identifying number of BEC, *x* (*m*, *t*) and *y* (*m*, *t*) are the two-dimensional matrix coordinates of BEC_*m*_ at time *t*, and *U*_*tn*_Δ*X* and *U*_*tn*_Δ*Y* are the variation components of BEC_*m*_ in the *X* and *Y* directions at time *t*, respectively.

### 2.4. Risk Analysis

For the purpose of this study, we used the modified Wells-Riley equation (equation (6) which was proposed by Rudnick and Milton [19]) to calculate the probability of infection risk for a susceptible population during evacuation in platform spaces:

(6) $$\begin{array}{c} P=1-\exp\left\{-\frac{iqpt}{Q}\times \left[1-\frac{V}{Qt}\left(1-\exp\left(-\frac{Qt}{V}\right)\right)\right]\right\}, \end{array}$$

where *P* is the probability of infection risk of susceptible individuals, *Q* is the outdoor air supply rate (m^3^/h), *V* is the volume of the ventilated space (m^3^), *i* is the number of infected people, *t* is the total exposure time (h), *p* is the breathing rate per person (m^3^/h), and *q* is the quantum generation rate of an infected person (quanta/h).

Person-to-person transmission of infectious diseases takes place through the recirculated air in confined spaces [20]. Moreover, because passengers do not stop at the platform, but go to their destination, the number of passengers in a platform space changes with time until it drops to zero when the evacuation ends. Thus, the outdoor air supply rate consists of individual breathing exchange and outdoor air supply, given by the following expression:

(7) $$\begin{array}{c} Q=\frac{n_{t}p}{f}, \end{array}$$

where *f* is the fraction of indoor air that is exhaled breath and *n*_*t*_ is the number of susceptible individuals at time *t*.

By substituting equation (7) and equation (1) in equation (6) can be expressed as

(8) $$\begin{array}{c} P\left(t\right)=1-\exp\left\{-\frac{iqft}{n_{t}}\times \left[1-\frac{\sum_{i=1}^{n_{t}}\text{BEC}\left(t\right)f}{n_{t}pt}\left(1-\exp\left(-\frac{n_{t}pt}{\sum_{i=1}^{n_{t}}\text{BEC}\left(t\right)\cdot f_{i}}\right)\right)\right]\right\}, \end{array}$$

where *P* (*t*) is the probability of infection of susceptible passengers at time *t*.

We used the updated mathematical model shown in equation (9), taking into account the passengers' distribution of overcrowding when *i* = 1, to estimate the infection probability. The reproduction number for an infectious disease in station platform space (*R*_*A*_) is expressed as

(9) $$\begin{array}{c} R_{A}=\left(n-1\right)\times P\left(t\right), \end{array}$$

where *R*_*A*_ is the number of secondary infections that arise when a single infectious case is introduced into susceptible people in a confined environment.

## 3. Case Study

With the method to derive the airspace volume from the individual distribution of overcrowding, this simulation has studied the infection risk during evacuation. The case assumes an airborne transmission condition, which was chosen under the base parameters given in Table 1.

*f* is a ratio that alters with the number of people present [19]. As more people are present in a room space, so the difference between the indoor and outdoor CO_2_ levels increases, while the value of Ca remains fairly constant. Therefore, a simplified equation (10) is applied to calculate intake fractions of indoor air pollutants [23]. This correction applies only for continuous sources and only under the condition that concentrations are not substantially different when a person is present or not in a particular microenvironment.

(10) $$\begin{array}{c} f_{i}\approx f\frac{\bar{Q}}{V\bar{a}}. \end{array}$$

We specified times *t*_0_ and *t*_1_ as 0 and 20 s, respectively, for demonstration purposes. The passengers' movements continued during the evacuation on the platform from *t*_0_ to *t*_*n*_ with a walking speed of 0.36–2.01 m/s. The exposure time was *t*_*n*_. To quantify the infection risk of the passengers, we divided the platform space into a two-dimensional matrix with coordinate dimensions of 450 × 12 m for (*X*_max_, *Y*_max_), which encompass BEC (*Z* = 2.4 m).

Figure 4 shows the schematic of the simulation process: train departure (check in ticket, pass the platform, boarding) and train arrival (get off, pass the platform, check out ticket). By turning on or off different accesses and doors, which were used to guide the index passengers, the simulation process was designed to provide three evacuation modes:

- For mode A, aimed for 1000 departing passengers, two entrance stairs (NS1-NS2), two entrance escalators (NE1-NE2), and 20 departure carriage doors (DD1–DD20) were opened for evacuation
- For mode B, aimed for 1000 arriving passengers, two exit stairs (XS1-XS2), two exit escalators (EE1-EE2), and 20 arrival carriage doors (AD1–AD20) were opened for evacuation
- For mode C, simultaneously aimed for 500 departing and 500 arriving passengers, two entrance stairs (NS1-NS2), two entrance escalators (NE1-NE2), two exit stairs (XS1-XS2), two exit escalators (EE1-EE2), 20 departure carriage doors (DD1–DD20), and 20 arrival carriage doors (AD1–AD20) were opened for evacuation

## 4. Results

### 4.1. Ventilated Volume

Figure 5 shows the relationship between the volume of the ventilated space and the exposure time of the passengers in the evacuation. Although all cases were set in the same station platform, the results were related to the evacuation modes and quite different from each other. The ventilated volumes reached a maximum of 5255 m^2^ at 540 s, 2334 m^2^ at 320 s, and 7996 m^2^ at 520 s under mode A, mode B, and mode C settings, respectively.

Figure 6 shows the individual distribution of overcrowding in mode C at 0, 20, 40, 100, 200, 400, and 600 s using Pathfinder. The stereo area occupied by the passengers gradually became larger and eventually stabilised as the time extended. The passengers were overcrowded near the stairs (XS1-XS2) and escalators (EE1-EE2) for a while.

### 4.2. Exposure Time

Figure 7 shows the relationship between the number of susceptible individuals and the exposure time for each given case. The exposure time of mode A, mode B, and mode C was 660, 400, and 680 s, respectively. Hence, overcrowding contributes to the exposure time in the three modes. The maximum number of susceptible individuals per unit time was 208 at 240 s, 427 at 60 s, and 472 at 80 s in mode A, mode B, and mode C, respectively. Evidently, the number of people clustered in model A per unit time is less and more uniform compared with that in other models.

### 4.3. Infection Risk

With the above results, the infection risk can be estimated by equation (9) and shown in Figure 8. In mode A, the risk increased as the time extended, peaked at *R*_*A*_ = 0.361 at 380 s, and then declined along the extending of time between 380 and 660 s. In model B, the risk increased as the time extended, peaked at *R*_*A*_ = 0.186 at 180 s, and then declined along the extending of time between 180 and 400 s. In model C, the risk increased as the time extended, peaked at *R*_*A*_ = 0.259 at 400 s, and then declined along the extending of time between 400 and 680 s. Hence, the median of risk in mode A is the highest, and the median of risk in mode B is the lowest.

## 5. Discussion

This study can provide further insights to observe the relationship between overcrowding in a platform space and the infection risk. It also examines differences of the infection risk in a station platform environment by varying the evacuation traces. As such, we have two major findings. First, the infection risk, especially during overcrowding, is quite different (Figure 8) in each case of the exposure scenario under a constant quantum generation rate. The building science model provided more data of the volume of the ventilated space (Figure 5), which was the primary vector for airborne infections. Moreover, controlling the number of susceptible individuals per unit time by strengthening guidance on the platform is more likely to reduce the risk of infection disease transmission. Second, departing passengers are at a lower risk of becoming infected than arriving passengers during an evacuation. Departing passengers, who are less overcrowded in the platform space than the arriving passengers (Figure 7), had a direct connection with the findings in the simulation.

Our study has several strengths. Many risk analyses of infection disease transmission used deterministic mathematical models [11, 15, 24, 25], but our study was based on Pathfinder, which simulated a dynamic overcrowding process. By contrast, many other studies that estimated the infection risk were performed without an analysis susceptible to individuals' spatial distribution. Here, we measured the trajectory area of all passengers from three modes to successfully solve the contradiction between the uneven spatial distribution of passengers and completely mixed air mentioned in the Wells-Riley model assumption (Figure 3). Finally, we are the first to apply Pathfinder (Figure 6) to calculate the infection risk in a station platform space.

In this simulation, our model does not allow the quantum generation rate and breathing rate per person changing with time. All exposed individuals were equally susceptible. As passenger position in the transport vehicles is fixed, passenger transport vehicles docking on the platform are outside the scope of the study. Notably, passengers have differential risks in the three modes (Figure 8). The risk of airborne transmission is greatest during passenger departure, whereas the risk of airborne transmission during passenger arrival is the lowest. Intuitively, one would presume that the risk of airborne transmission is greatest when passenger departure and arrival simultaneously occur in a platform space. We attribute these counterintuitive findings to the differences in the evacuation flow of passengers on the platform.

Interestingly, the results of coupling building science model and the Wells-Riley model were more accurate than those of the standard model, where the ventilated volume within the Wells-Riley model was assumed as the room volume [26].  Figure 9 shows the relationship of *R*_*A*_ between the standard model and the optimised model. There are two main differences:

- The range of *R*_*A*_ obtained by the standard model is obviously higher than the optimised result of mode A, mode B, and mode C
- *R*_*A*_ will show ups and downs over time as the number of passengers on the platform gradually decreases during an evacuation. By contrast, the standard model cannot reflect this from numerical changes.

Although we have identified differential risks for passengers in the platform space depending on the evacuation modes, the study has several limitations. First, the study only selected the simplest type of station platform, not including complex passenger paths, such as business, leisure, and entertainment, and the number of passengers in the study setting was limited to extreme situations. Second, this simulation is not suitable for interventions using personal protective equipment or improving ventilation to observe its impact on the risk of airborne transmission. Third, no further research was made on the effect of the degree of overcrowding on host susceptibility.

## 6. Conclusion

In summary, we provided a framework to quantify the risk of airborne transmission with overcrowding in confined spaces, especially the dynamic distribution of individuals, by coupling building science model and the Wells-Riley model, and to estimate the likelihood of an outbreak when an index case is introduced into a susceptible population and associated with various evacuation settings. Our results reinforce the importance of a correlation between overcrowding and the risk of airborne transmission in developing engineering or administrative solutions to artificially minimise the spread of airborne infection in platform spaces.

## Figures and Tables

**Figure 1:** Three-dimensional station platform with a dimension of 450 × 12 × 4 m as the base condition space.

**Figure 2:** (a) Basic exposure cell; (b) room space; (c) volume of the ventilated space.

**Figure 3:** (a) Passengers' distribution of overcrowding; (b) trajectory of each individual; (c) volume of the ventilated space.

**Figure 4:** Schematic of the simulation process: train arrival and train departure.

**Figure 5:** Relationship between the volume of the ventilated space and the exposure time of the passengers during evacuation.

**Figure 6:** Individual distribution of overcrowding in mode C.

**Figure 7:** Relationship between the number of susceptible individuals and the exposure time for each given case.

**Figure 8:** Infection risk estimated by equation (9).

**Figure 9:** Relationship of *R*_*A*_ between the standard model and the optimised model.

**Table 1:** Base parameters used to estimate the infection probability, taking into account the variation of individual distribution.

Variable	Parameter	Value
Number of susceptible individual	*n*_*t*_	From simulation
Volume of shared airspace (m^3^)	∑_*i*=1_^*n*_*t*_^BEC_*i*_(*t*)	From simulation
Total exposure time (h)	*t*	From simulation
Breathing rate (m^3^/h)	*p*	0.3^a^
Quantum generation rate (quanta/h)	*Q*	67^b^
Fraction of indoor air exhaled by infected people	*f*	0.0306^c^
Number of infected people	*i*	1

^a^Cited from [21]. ^b^Cited from [22]. ^c^Cited from [15].

## Data Availability

The datasets used and/or analyzed during the current study are available from the corresponding author upon request.
